# Anti-inflammatory and protective investigations on the effects of Theranekron® ”an alcoholic extract of the Tarantula cubensis” on wound healing of peritoneal in the rat: an in vivo comparative study

**DOI:** 10.1186/s13000-015-0252-x

**Published:** 2015-04-02

**Authors:** Farajollah Adib-Hashemi, Farshad Farahmand, Shamim Fattah Hesari, Bijan Rezakhaniha, Ehsan Fallah, Amir Farshid Fayyaz, Masoomeh Dadpay

**Affiliations:** Department of Clinical Science, Faculty of Veterinary Medicine, Tehran University, Tehran, Iran; Graduated, Faculty of Veterinary Medicine, Garmsar Branch, Islamic Azad University, Garmsar, Iran; Orthopedic Surgeon, Department of Surgery, Imam Reza hospital, Tehran, Iran; Department of Urology, Imam Reza Hospital, Tehran, Iran; Department of Orthopedic and Trauma Surgery, AJA University of Medical Sciences, Tehran, Iran; Departmen of Legal Medicine, AJA University of Medical Sciences, Tehran, Iran; Department of Pathology, Imam Reza Hospital, AJA University of Medical Sciences, Tehran, Iran

**Keywords:** Theranekron, Histopathology, Wound, Regeneration, Rat

## Abstract

**Background:**

The present study sought to investigate the effects of Tarantula cubensis extract (TC; Theranekron®) on the histopathological scores of peritoneal wound healing after laparotomy in the rats.

**Methods:**

This study was designed to investigate the effects of Theranekron on the peritoneal wound healing after wound creation, on days9, 14, 19, 24 and 29 post-injury in rats. Twenty-four mature Wister-albino male rats were randomly divided into two groups. In the experimental group, TC was repeatedly injected subcutaneously (SC) over the lesion 9, 14,19 and 24 days after laparotomy, whereas the control group received only normal saline by subcutaneous injection and then the animal groups were euthanized9, 14, 19, 24, and 29 days after wounding respectively by intravenous injections of pentobarbital (50 mg/kg). Finally, assessment of the peritoneal wound healing between the groups was carried out by histopathologic data and statistical tests as Mann-Whitney U, Wilcoxon W and Z

**Results:**

Histopathological examination indicated significant improvement in angiogenesis, re-epithelialization and less inflammatory response in comparison to control and also, revealed matured, compact and parallel deposition of collagen fibrils on day 29. So, at long term, treatment reduced the inflammation and increased the quality and rate of wound re- epithelialization compared to controls(P < 0.05). Furthermore, excluding the control group, rats exhibited the most pronounced effect on wound closure, with the statistically significant improvement in wound healing being seen at post-operative day 29. Moreover, collagen content on days 24 and 29 in the test group was found to be higher than in the healthy group. To warp up, treated groups had a significant increase in peritoneal wound healing area compared to the control group on all days (P < 0.05).

**Conclusions:**

Our results suggested that Theranekron have delivered a novel therapeutic route for wound treatment in clinical practice.

**Virtual slides:**

The virtual slide(s) for this article can be found here: http://www.diagnosticpathology.diagnomx.eu/vs/2958770714954315.

## Background

Peritoneal wounds usually occur following trauma, ablation of malignancy of the genitalia, low pelvic tumors, or following thermal or electrical injuries. These wounds remain a significant problem and can commonly present as wound infection, abscess, dehiscence, delayed healing, or persistent peritoneal sinuses. These wounds result in significant morbidity requiring prolonged hospital stay, hospital readmission, home-nursing wound care needs; all involving significant medical costs [1].

Healing of the wound is a dynamic and complex process and the clinical evaluation of its early and late phase may include biochemical [2,3], immunological [4], histopathological [5] and mechanical [6,7] studies. In healing, after cessation of bleeding (hemostasis) and clot formation, the process can be divided into three overlapping phases: inflammation, proliferation and scar maturation. In general, injury is accomplished by fibroplasia, angiogenesis and migration of fibroblasts, endothelial cells and epithelial cells lead to wound contraction [8]. The healing process starts with the formation of granulation tissue and ends with scar formation. The degree of wound healing is determined by inflammation [9], a vital and protective response offered by the injured cells at wound site that actually starts the process of tissue repair [10].

Treatment methods that allow wounds to heal faster and minimize cosmetic defects and the production of exuberant granulation tissue are the most appropriate [11-13]. In parallel, Theranekron® (Richter Pharma, Wels, Austria) is an alcoholic extract of the venom of Tarantula cubensis, which remains active in pharmaceutical compounds for a considerable time. Many systemic effects were described for Theranekron such as antiphlogistic, demarcative, necrotizing action [14], but there are few reports of Theranekron effects on wound healing in farm animals [14-16].

On the other hand, TC (Figure 1A). has been used in homeopathy to treat mixed mammary tumors, pododermatitis abscesses with burning pains, gangrene, septicemia and toxemia by forming a demarcation line around the lesions [17-19]. In addition, TC reduced inflammation and tarsal bursitis volume, stimulated epithelialization in the full thickness cutaneous wounds [15,20], improved the uterine involution, and treated the genital microbial diseases [21], oral ulcers [20], and cutaneous papillomatosis of various species of animals. The aim of this study was to evaluate of the effects of theranekron on the peritoneal wound healing based by histopathological features.

**Figure 1:** **Operations/Surgical Procedures. A**: Tarantula cubensis (Cuban Spider) and Theranekron is a homeopathic remedy prepared from the spider Tarantula *.* **B**: Laparotomy and exposure of the peritoneal cavity and two buttons created of the abdominal wall. **C**: Note that the peritoneal and partially of the muscle was closed by purse string suture. **D**: The abdomen was closed in two layers by silk sutures (with separate vicryl 3/0 stitches for the musculoperitoneum and avicryl 3/0 running suture for the skin).

## Methods

### Animals welfare

All experimental protocols were approved by the local animal care committee in accordance with Faculty of Garmsar Veterinary Medicine office regulations. The animals were kept two by two in individual propylene cages under standard laboratory conditions by the dimensions of 30 × 50 × 25 cm^3^. Rats were maintained on a 12 hour light/dark cycle at 22 ± 1°C and 50 ± 10% humidity. The animals were kept in standard room conditions and fed with standard rat diet and water ad libitum.

### Pharmaceutical ingredients

Theranekron® alcoholic extract (1:100) of Tarentula cubensis in alcoholic solution 1 mg/ml, purchased from Richter-Pharma AG, Wels, Austria, and or can be expressed that each ml of pharmaceutical ingredient Theranekron contains: 1.0 mg alcoholic extract (1:100) from Tarantula cubensis in alcoholic solution, and the final dilution was D6 and potentisation was performed according to method 4b of the European Homeopathic Pharmacopoeia [15,18,20,21].

### Experimental design and dose preparation procedure

In current study, 24 male Wister-albino rats, weighing 210–230 g, with averagely 4 weeks old were selected. The rats were divided into two groups and randomly allotted into one of two experimental groups each group contained 12 animals.

Control animals in group I received normal saline (a single dose 0.3 ml with intervals 5 days for 29 days, SC), and experimental animals in group II received Tarrantula cubensis extract (Theranekron, 1:100/D2, 0.3 ml, Richter Pharma, Austria) following surgery. On days 9,14, 19, 24 and 29 after injury, the same volume of TC extract with dose 0.3 ml was injected subcutaneously at the site of injury in the injured experimental group at the same time with intervals 5 days for 29 days. Clinical signs of rats of both groups were recorded during day 9, 14, 19, 24 and 29 of treatment.

### Surgical procedure

Anesthesia was achieved with subcutaneous administration of 75 mg/kg ketamine HCl and 10 mg/kg xylazine HCl. Laparotomy was performed through a 3-cm midline incision. The abdomen was shaved, prepared and disinfected with1% iodine alcohol and then, abdominal cavity was entered via a 3 cm vertical midline incision. Then with peritoneal cavity exposure two buttons were made of the abdominal wall and with this method (Figure 1B and C), the remaining tissue between buttons is caused necrosis by anemia or congestion. The abdomen was closed in two layers by silk sutures (with separate vicryl 3/0 stitches for the musculoperitoneum and avicryl 3/0 running suture for the skin) (Figure 1D). A mixture of iodine and oxytetracycline was sprayed to the laparotomy site as an antibiotic agent and especially due to its bitter taste, it inhibited rats to chew the sutures and prevent evisceration.to warp up, the wound tissue was removed from control and experimental rats by sacrificing the animals on the 9, 14, 19, 24, and 29 days and or another definition, with interval 5 days,the animal groups were euthanized 9,14, 19, 24, and 29 days after wounding respectively by intravenous injections of pentobarbital (50 mg/kg).

### Histopathological examination

The wounded tissues with 2X2 cm piece of parietal peritoneum, underlying muscle and peripheral unwounded skin were harvested, pinned on a plastic plate (to keep the tissue flat) and fixed in 10% buffered formalin. After fixation, each sample was cut into 3 pieces. All pieces were embedded together into a paraffin block, and 5 μm-thick histological sections were obtained and after wound creation and the abdominal wall were harvested and underwent histologic evaluation. Two pathologists examined all representative fascia sections in each rat histologically under a light microscope in blinded fashion.

### The scoring system used for histological examination

All specimens were evaluated individually by two histologists who were blinded to the drug type and the time from wounding. The main histologic outcome measures included the amount of inflammatory infiltrates for extent and severity, fibroplasia, collagen deposition, neovascularization (angiogenesis), re-epithelialization or complete repair. The Abramov’s histologic scoring system was used for this study [22]. Abramov’s system assessed each parameter independently and assigned a score of 0–3. inflammatory infiltrates or extent, collagen deposition and complete repair were graded as: 0 (none), 1(scant), 2 (moderate), 3 (abundant).and also, severity of inflammation was scored as follows: 0 – no inflammation; 1– presence of giant cells, occasional lymphocytes and plasma cells; 2 – presence of giant cells, plasma cells, eosinophils and neutrophils; and 3 – presence of many inflammatory cells and microabscesses. The amount of fibrosis was scored as: 0 = no fibrosis; 1 = minimal, loose; 2 = moderate; and 3 = florid dense. The fibroblast maturation or fibroplasia of granulation tissue was graded as: 0 (immature), 1 (mild maturation), 2 (moderate maturation), 3 (fully matured). Neovascularization was graded as: 0 (none), 1(up to two vessels per high-power field [HPF]), 2 (3–4 vessels per HPF), 3 (more than 4 vessels per HPF).

### Statistical analysis

For statistical analysis, Mann-Whitney U, Wilcoxon W, Z and the asymptotic significance (2-tailed) were performed to analyze the significant differences between groups and a statistically significant difference was considered at the level of P < 0.05.

## Results

### Clinical observations

The affected rats manifested clinical sings of appetite loss, fever, weakness, apathy and /or tiredness, while no clinical signs were observed in the control groups, and also, at all stages of the experimental, after laparotomy , the formation of intraperitoneal adhesion in the location of button was a constant finding in both groups (Figure 2). Furthermore, wound areas decreased rapidly in size between days 24 and 29 in both the test and control groups

**Figure 2:** **Note that adhesion sites in the location of buttons.**

### Histopathological findings

In regards to the histological outcomes from in vivo experiments, in the treated groups; on the 9rd day after the operation, there was a wound extending deep to muscle layer where the cells were edematous. The wound region was covered with low number of the inflammatory cells and the tissue was only lightly infiltrated with polymorphonuclear leukocytes, thus the inflammatory phase was almost finished together with moderate number of fibroblast and collagen matrix.

In control group, the increased amounts of mononuclear inflammatory cells such as macrophage, lymphocytes and its accumulation together with the presence higher of fibroblasts and low blood vessels were detected (Figure 3) (Table 1). Finally, in day9, the results of the histologic analysis showed that 95% of the severity and extent of inflammation and fibroplasia in the wound were significantly higher statistically in the experimental group compared with the control group (P < 0.05), also in other healing factors, no histologic difference were noted between the test and control groups (P > 0.05) (Figure 4) (Table 2).

**Figure 3:** **Day14: ConrolG: the high amounts of fibroblasts and the low of collagen together with the presence of the inflammatory cells accumulation,Day14:Experimental G: the formation of numerous blood vessels with the presence of mononuclear cells together with the moderate amounts of fibroblast and collagen matrix, Day19:ConrolG: The numerous number of the blood vessels (angiogenesis)and fibroblast compeer with the less amount of inflammatory cells, Day19:Experimental G: collagen deposition and fibroblast without blood vessels and reduced inflammatory cells infiltration, Day24:ConrolG: parenchymal fibroblast matrix patch induces angiogenesis and increases fibroblasts, Day24:Experimental G: increased collagen deposition together with drastic reduction of inflammatory cells, Day29:ConrolG: collagen deposition and fibroblasts are seen , Day24:Experimental G: Reconstruction of full-thickness defects with thick collagen matrix without angiogenesis and inflammation cells.**

**Table 1:** **Evaluation of histological scoring system described by Abramov’s in the control and experimental groups on the peritoneal wound healing in the rats**

**histological scores**	**Day 14**		**Day 19**		**Day 24**		**Day 29**	
	**control group**	**experimental group**	**control group**	**experimental group**	**control group**	**experimental group**	**control group**	**experimental group**
The extent of inflammation	+++	+	++	^_^	+	^_^	^_^	^_^
The severity of inflammation	+++	+	+	^_^	+	+	+	^_^
Angiogenesis	+++	+++	+++	++	+++	^_^	++	^_^
Fibroplasia	+	++	+	++	++	++	+	+++
Complete re-epithelialization or complete wound healing	+	+	+	++	++	++	+	+++

The number of the histopathological scores: 0:^_^; 1:+; 2:++; 3:+++.

**Figure 4:** **Histopathological scores in all days of the experimental.** CG: Control Group, EG: Experimental Group. Series1: The extent of inflammation*,* Series2: **T**he severity of inflammation, Series3: Angiogenesis, Series4: Fibroplasia, Series5: **C**omplete wound healing.

**Table 2:** **Analysis of histological scores by test statistics**

**Histological scores**	**Day 14**				**Day 19**				**Day 24**				**Day 29**			
	**MWU**	**Wilcoxon W.**	**Z test**	**Asymp. Sig. (2-tailed)**	**MWU**	**Wilcoxon W.**	**Z test**	**Asymp. Sig. (2-tailed)**	**MWU**	**Wilcoxon W.**	**Z test**	**Asymp. Sig. (2-tailed)**	**MWU**	**Wilcoxon W.**	**Z test**	**Asymp. Sig. (2-tailed)**
The extent of inflammation	0.000	10.000	−2.494	0.013	0.000	10.000	−2.494	O.O13	0.000	10.000	−2.646	0.008	6.000	27.000	−2.345	0.019
The severity of inflammation	0.000	10.000	−2.646	0.008	0.000	10.000	−2.646	0.008	8.000	18.000	0.000	1.000	6.000	27.000	−2.345	0.019
Angiogenesis	4.000	14.000	−1.528	0.127	0.000	10.000	−2.646	0.008	0.000	10.000	−2.494	0.013	0.000	21.000	−3.146	0.002
Fibroplasia	0.000	10.000	−2.494	0.013	0.000	10.000	−2.646	0.008	4.000	14.000	−1.528	0.127	0.000	21.000	−3.146	0.002
complete wound healing	8.000	18.000	0.000	1.0000	0.000	10.000	−2.646	0.008	4.000	14.000	−1.528	0.127	0.000	21.000	−3.317	0.001

MWU: Mann–Whitney U, Asymp. Sig. (2-tailed): Asymptotic Significance (2-tailed).

On the day 14 of treatment group, there’s absence of wound regeneration with minimal neovascularization and cellular infiltrates and also, dilated blood vessels with stasis were seen underneath and in the granulation tissue. Moreover, thick coarse collagen fibers accumulated in the wound region under the granulation tissue with cellularity increases mainly due to fibroblasts proliferation and new matrix deposition.

In control group, the low amounts of inflammatory cells together with the presence higher of fibroblasts and angiogenesis were found (Figure 3) (Table 1). Finally, in day14, in all wound healing factors, no significant differences were observed histologically in 95% of both groups (P > 0.05) (Figure 4) (Table 2).

On the days 19 and 24 of treatment group, inflammatory cells are few and are mainly mononuclear cells (lymphocytes, plasma cells and macrophages) and these cells remain at the border of the scar. At this time point a small number of myofibroblasts and luminized vessels were present in the granulation tissues of wounds. And compared to the first two groups, healing was better. The surface was completely covered with epithelium. Compared to other groups, less scar tissue formation was noted with thick and almost normally arranged collagen fibers with the number of mild to moderate fibroblasts.

In control group, the presence of high numbers of fibroblasts, collagen and angiogenesis were observed (Figure 3) (Table 1). Finally, in days 19and 24, significant differences were observed histologically in 95% of both groups on the extent of inflammation and angiogenesis (P < 0.05), also in other healing factors, no histologic difference were noted between the test and control groups (P > 0.05) (Figure 4) (Table 2).

In the experimental group, on the 29th day, histopathology revealed that decreased inflammatory cell infiltration, the fibroblasts became increasingly mature and collagen deposited. Furthermore, the results of the histologic analysis showed that the collagen deposition in the wound was significantly higher compared with the other groups and also, the inhibition of angiogenesis was observed.

In control group, the low number of fibroblasts together with collagen matrix and angiogenesis were observed (Figure 3) (Table 1). Finally, in day 29, significant differences were observed histologically in 95% to 99% of both groups (P < 0.05) (Figure 4) (Table 2).

## Discussion

In the present study, the wound healing process of rat peritoneal was histopathogically described during the first twenty-nine days. Other studies evaluated histologically only certain time intervals, i.e. the seventh day by Menetrey et al. [23], the fourth and seventh day by Rasik et al. [24], the second, fourth, seventh and fourteenth day by Whelan et al. [25] and the first, third, fifth, seventh and tenth day by Connolly et al. [26] and they observed an influence of various factors on the wound healing. Our study correlates with other studies researching histopathologically the wound healing process (per primam intentionem) of the rat skin [27-33]. The most significant pathological changes occur during the first fourteenth days of wound healing [34] and this contributes to the importance of our study. And in the present study, the tissue samples taken from the wounds were examined histopathologically for inflammatory cell infiltration, fibroblast activity, granulation, vascularization and re-epithelialization or complete regeneration. These assessments were performed on 14 th, 19 th, 24 th and on the 29 th day after wounding.

Wound healing is complex and involves multiple molecular processes, including inflammation, angiogenesis, granulation tissue formation, re-epithelialization, and wound contraction [35] .In the tissue repair process, inflammatory cells promote the migration and proliferation of endothelial cells, leading to neovascularization of connective tissue cells which synthesize extracellular matrices including collagen, and of keratinocytes resulting to re-epithelialization of the wounded tissue [5,10,15,32]. Inflammation, collagen maturation, and scar formation are some of the many phases of wound healing, which run concurrently but independent of each other

In our study, the complete regeneration of the peritoneal wound was finished on the first twenty-nine day after the surgery, which is comparable to humans [35,36]. In a study, Sardari et al., [15] reported that Theranekron can significantly stimulate epithelialization in full thickness wounds in cows during the first 14 days of healing and this is partially in agreement with our results, because in the present study complete epithelialization was observed in the 29th day. Our results showed that fourteenth days post-surgery allow evaluating the low amounts of the inflammatory reaction and the beginning of re- epithelialization. Twenty-nine days are suitable for the assessment of the proliferative phase and re- epithelialization as well. Finally, twenty-nine days after surgery is possible to evaluate wound maturation and scar formation.

Some reports have described Theranekron as having beneficial effects on the healing of cow hoof injuries [14]. In parallel ,in the present study, significant differences was observed in peritoneal wound healing in the test and control groups (P < 0.05). Furthermore,in a study with therankron, oryan et el., [37]. showed the anti-inflammatory effects of Tarantula cubensis (theranekron) on the tendon lesions and the number of the inflammatory cells and the amounts of tissue swelling in the injured treated tendon was significantly lower than the injured control tendons.This is in agreement with our study, was observed that the anti-inflammatory effects of theranekron on the peritoneal wound healing in rat and also, detected that the amounts of the inflammatory cells the experimental groups were significantly lower than the injured control groups (P < 0.05).

To our knowledge, the present study is the first to reveal that subcutaneous administration of theranekron accelerates peritoneal wound healing using rat wound model. It was demonstrated by a significant increase in the rate of wound closure and enhanced epithelialization. A significant increase (P < 0.05) in collagen levels were also observed, which was further supported by histopathological studies and gain in granuloma angiogenesis. Collagen and angiogenesis are required for normal wound healing. Therefore, stimulating their synthesis when wound repair is defective would be beneficial for promoting wound healing. And also, collagen is produced by fibroblasts and helps the wound gain tensile strength during repair [38]. Several studies reported an increase in wound tensile strength, which depends on factors in addition to collagen deposition, namely matrix deposition and cell migration [39]. In the beginning a wound will only have little breaking strength because the clot will alone be holding the edges together [40,41]. Thereafter tensile strength increases rapidly as collagen deposition increases and cross-linkages are formed between the collagen fibres. Our results also showed theranekron treatment caused a significant increase in wound collagen content measured as H&E staining.

Angiogenesis is a complex, multistage process, in which a variety of cells are involved in the construction of new blood vessels [42-44]. In the present study, as healing progressed, these vessels decreased in number, but were noted to be larger calibre mature blood vessels at day 14 in theranekron treated group compared with control group, which were consistent with this previous study [45].

## Conclusions

This study demonstrated that histopathological evaluation of the wound site provided evidence of a more desirable histological organization of the tissue in response to theranekron treatment. Treatment of rats with theranekron resulted in an enhancement of wound healing, as evidenced by increased wound re-epithelialization closure, fibroblasts and the formation of new blood vessels. The results of our study show the efficacy of theranekron treatment on wound healing in animals. On the basis of these results, we believe that theranekron is a therapeutically beneficial method to treat wounds in clinical practice.
